The article "Diagnostic Value of Ultrasonography Combined with Hysteroscopy in Intrauterine Space-Occupying Abnormalities" was published in 2022. Journal: Contrast Media Mol Imaging.

# Diagnostic Value of Ultrasonography Combined with Hysteroscopy in Intrauterine Space-Occupying Abnormalities

**DOI:** 10.1155/2022/6192311

**Published:** 2022-08-30

**Authors:** Zongbao Xia, Hong Jin

**Affiliations:** ^1^Department of Gynaecology, Jingmen First People's Hospital, Jingmen 448000, Hubei, China; ^2^Department of Ultrasound, The First People's Hospital of Jingmen, Jingmen 448000, Hubei, China

## Abstract

The aim of this study was to analyze the diagnostic significance of ultrasonography combined with hysteroscopy for intrauterine space-occupying abnormalities. A total of 99 patients with uterine space-occupying abnormalities treated in hospitals were enrolled. The patients were divided into three groups according to different disease types: the submucosal myoma group, endometrial polyp group, and placenta residue group, with 33 patients in each group. The differences and diagnostic effects in intrauterine ultrasound, hysteroscopic findings, and surgical histopathology were observed in each group. Outcome measures: it was to compare the sensitivity, specificity, and accuracy of intrauterine ultrasound and angiography for intrauterine space-occupying lesions using surgical and pathological examination methods as the gold standard; the relationship between the location, number, size, appearance, and serosal layer of intrauterine lesions was clearly shown; the location, number, appearance, and echogenicity of space-occupying abnormalities under hysteroscopy were observed. The results showed that the diagnostic rates of endometrial polyps, submucous myoma, and residual placenta were 90.9%, 80.8%, and 72.7%, respectively. However, the sensitivity, specificity, and accuracy of ultrasonography in the diagnosis of endometrial polyps were 90.0%, 66.7%, and 87.9%, respectively; those of hysteroscopy in the diagnosis of endometrial polyps were 96.7%, 66.7%, and 93.9%, respectively; and combined diagnosis was 96.7%, 100.0%, 97.0%, 100.0%, and 75.0%. The sensitivity, specificity, and accuracy of ultrasonography in the diagnosis of submucous myoma of the uterus were 88.9%, 50.0%, and 81.8%, respectively; those of hysteroscopy in the diagnosis of submucous myoma of the uterus were 96.3%, 83.3%, and 93.9%, respectively; and combined diagnosis was 100.0%, 83.3%, 97.0%, 96.4%, and 100.0%. The sensitivity, specificity, and accuracy of ultrasonography in the diagnosis of uteroplacental remnants were 87.5%, 66.7%, and 81.8%, respectively; those of hysteroscopy in the diagnosis of uteroplacental remnants were 91.7%, 77.8%, and 87.9%, respectively; and combined diagnosis was 95.8%, 88.9%, 93.9%, 95.8%, and 88.9%. In summary, ultrasonography combined with hysteroscopy can improve the diagnostic sensitivity and accuracy for intrauterine space-occupying abnormalities.

The article "Diagnostic Value of Ultrasonography Combined with Hysteroscopy in Intrauterine Space-Occupying Abnormalities" was published in 2022. Journal: Contrast Media Mol Imaging.

## 1. Introduction

Transvaginal ultrasound combined with sonohysterography (SHG) is to place contrast agent (generally without bacterial saline) through the cervix into the uterine cavity, manually dilate the uterine cavity, and then separate the endometrium, and transvaginal sonography (TVS) should be performed to timely monitor the endometrial condition and intrauterine problems [1]. SHG has been a commonly used clinical diagnostic method in recent years and belongs to the method of noninvasively detecting intrauterine lesions, which enhances the diagnostic sensitivity and specificity of endometrial diseases [2]. Studies have confirmed that SHG has a high clinical value for this disease when patients present with diffuse or focal intrauterine lesions [3]. Contrast-enhanced ultrasound can clearly observe whether the patient's lesions are diffuse or local and can also clearly show the location, size, number, shape, and other characteristics of focal lesions, thus further enhancing the sensitivity and specificity of diagnosis [4]. Contrast-enhanced ultrasound belongs to transabdominal ultrasound monitoring technology, which is affected by obesity and other problems due to needing a full bladder for patients during the detection process, which limits the clinical application of this technology [5]. TVS does not require a full bladder, and is not affected by obesity and gas in the intestine, so the high-frequency probe can clearly show the structural changes of the uterus, ovary, and surrounding tissues [6]. Intrauterine space-occupying abnormalities include endometrial polyps, endometrial hyperplasia, submucous myoma, residual embryos, and endometrial cancer, with endometrial polyps and submucous myoma being the most common [7]. Intrauterine disease is a common gynecological disease, which is generally characterized by menstrual dripping, prolonged menstruation, and irregular vaginal bleeding [8]. Because the etiology of intrauterine disease is complex and the nature is difficult to define, early and definitive clinical diagnosis is conducive to the development of appropriate treatment options [9].

Intrauterine lesions such as submucous myoma, endometrial polyps, endometrial hyperplasia, and endometrial cancer are the main factors of paradoxical uterine bleeding before and after menopause [10]. The main features of SHG images of intrauterine lesions are as follows: endometrial hyperplasia, often showing features of diffuse thickening of the endometrium is mainly diagnosed and classified using curettage and pathological examination [11]. Endometrial polyps, which mainly show hyperechoic mass adhesions of the uterine wall with smooth margins, and mostly present oval structures, but also conical, rod-shaped or shuttle-shaped, irregular shapes, and the upper end of the pedicle can flow with the presence of contrast agents [12]. Submucous myomas of the uterus, which mainly show spherical or hemispherical structures and protrude in the uterine cavity, are mostly characterized by a wide base, hypoechoic or isoechoic, and swing without the influence of contrast agents [13]. The uterine cavity was deformed, and some endometrial hyperechoic lines could be seen entangled on the surface of the fibroid protrusion, with a smooth front and disappearance of endometrial hyperechoic lines at the base [14]. Hysteroscopy is an emerging field that appears in the field of modern gynecology, and it is a product combining electro-optic, ultrasound, and medical treatment [15]. Hysteroscopic techniques include hysteroscopic detection, treatment, and surgery [16]. Hysteroscopy can observe the physiological and pathological development in the uterine cavity and has become the most important diagnostic method for gynecological diseases, especially intrauterine bleeding diseases [17]. It has deep clinical value in the diagnosis and treatment of space-occupying abnormalities in the uterine cavity, especially in the pretreatment evaluation of hysteroscopic surgery [18].

The article "Diagnostic Value of Ultrasonography Combined with Hysteroscopy in Intrauterine Space-Occupying Abnormalities" was published in 2022. Journal: Contrast Media Mol Imaging.

In order to investigate the diagnostic value of ultrasonography and hysteroscopy for intrauterine space-occupying abnormalities, patients with intrauterine space-occupying abnormalities were studied to compare and analyze the diagnostic values of ultrasonography and hysteroscopy for this disease, providing research data for improving the clinical diagnostic effect of intrauterine space-occupying abnormalities.

## 2. Materials and Methods

### 2.1. Study Subjects

Ninety-nine patients with uterine space-occupying abnormalities treated in hospitals from February 2019 to February 2020 were enrolled. According to the lesions, they were divided into submucosal myoma (submucosal myoma group), endometrial polyp (endometrial polyp group), and placenta residue (uterine placenta residue group) groups, with 33 patients in each group, aged 17–41 years, with an average age of (31 ± 2.63) years. All cases were confirmed by pathological examination. This study was approved by the ethics committee of the hospital, and the families of patients signed the consent form.

Inclusion criteria: Patients were diagnosed with submucous myoma or endometrial polyps or residual placenta; patients aged over 16 years old. The patient has some ability to understand and express. The consent of the subjects and their families was obtained. Exclusion criteria: patients with serious mental illness. The patient developed serious complications. The patient had a long history of substance abuse.

The article "Diagnostic Value of Ultrasonography Combined with Hysteroscopy in Intrauterine Space-Occupying Abnormalities" was published in 2022. Journal: Contrast Media Mol Imaging.

### 2.2. Imaging Examination

Color Doppler ultrasound equipment was used. the probe was a vaginal probe with a frequency of 5.0 ∼ 7.5 MHZ. In addition to patients with uterine fetal residues, other patients underwent vaginal ultrasound examination at 3 ∼ 6 days after menstruation. The vaginal probe was disinfected first. After disinfection, the probe was inserted into the double-chamber angiography tube from the cervix, and 5.0 mL of normal saline was injected into the balloon. The balloon was placed at the cervix, and then the vaginal probe was placed. The uterine cavity was filled with 20 mL saline. The location, shape, size, and echo characteristics of the lesions were observed and recorded. After the examination, a 4-day follow-up was conducted and antibiotics were routinely used for anti-infective treatment.

A high definition hysteroscopic camera system（Image I HD）was used. The balloon catheter was inserted into the cervix one day before hysteroscopy, and 2 misoprostol was embolized by vagina, or 2 misoprostol was taken orally 3–7 hours before operation. Hysteroscopy was inserted after cervical dilatation, 5.2% glucose was used as the medium of uterine dilatation, and the uterine pressure was controlled at 8.2–5.2 kPa. The uterine appearance, color, membrane thickness, adhesion status, uterine malformation, and tubal opening morphology of the patients were gradually analyzed. The diagnosis of the disease was based on the characteristics under hysteroscopy. For suspicious lesions, microscopic biopsy or pathological examination was needed to determine.

### 2.3. Outcome Measures

Surgical pathological examination methods were taken as the gold standard. Comparing the sensitivity, specificity, and accuracy of intrauterine ultrasound and angiography for space-occupying lesions in the uterine cavity can clearly show the relationship between the location, number, size, appearance, and serosal layer of uterine cavity lesions.

The location, number, appearance, echo, and other manifestations of space-occupying abnormalities under hysteroscopy were observed.

### 2.4. Statistical Analysis

The statistical analysis was completed using the SPSS 22.0 software. Measurement data were expressed as the mean ± standard deviation, and differences were compared using rank sum test. Enumeration data were expressed as frequency or percentage, and X^2^ test was used for difference comparison. *P* < 0.05 was considered statistically significant.

## 3. Results

### 3.1. Basic Data

The age of patients in the submucous myoma group was 17–39 years, with an average of 28.11 ± 1.82 years. The age of patients in the endometrial polyp group ranged from 19 to 41 years, with an average of 29.26 ± 2.68 years. The age of patients in the placenta residue group ranged from 23 to 34 years, with an average of 25.07 ± 2.54 years. After comparison, it was found that there was no significant difference in the basic data among the submucous myoma group, the endometrial polyp group, and placenta residue group (*P* > 0.055) (Table 1).

The article "Diagnostic Value of Ultrasonography Combined with Hysteroscopy in Intrauterine Space-Occupying Abnormalities" was published in 2022. Journal: Contrast Media Mol Imaging.

### 3.2. Image Analysis of Normal Uterine Cavity through Abdomen and Vagina

Figure 1 demonstrates a normal ultrasound image of the uterine cavity. Endometrium was detected by transabdominal ultrasound. The main characteristics were various degrees of thickening or mass-like slightly low or some high echo, and the basal part of the surrounding boundary cannot be distinguished. The endometrium of TVS was mainly characterized by various degrees of thickening or mass-like echoes, with clear boundaries, which can be used for location judgment and cannot effectively determine multiple lesions. SHG can show the size of dilated uterine cavity, and the shape of uterine cavity was different, without echo area. It can clearly show the edge, location, number, and width of base of the lesion.

### 3.3. Comparison of Diagnostic Value of Ultrasound and Hysteroscopy in Endometrial Polyps

The diagnostic value of ultrasonography and hysteroscopy in endometrial polyps was compared. Single or multiple intrauterine synapses can be clearly seen in the ultrasound images and hysteroscopy images of patients with endometrial polyps, and their shape is cylindrical or bamboo shoot-tip, mainly medium or high-intensity echo. Liquid flow can be observed in the fluid of individual polyps (Figure 2).

The pathological diagnosis of 30 patients with endometrial polyps after operation was confirmed in 33 cases (90.9%). Twenty-seven cases of endometrial polyps were diagnosed by uterine ultrasound, and the diagnostic sensitivity, specificity, accuracy, positive predictive value, and negative predictive value were 90.0%, 66.7%, 87.9%, 96.4%, and 40.0%, respectively. Hysteroscopy was used to diagnose 29 cases of endometrial polyps, with diagnostic sensitivity of 96.7%, specificity of 66.7%, accuracy of 93.9%, positive predictive value of 96.7%, and negative predictive value of 66.7%. The combined diagnostic sensitivity was 96.7%, specificity was 100.0%, accuracy was 97.0%, positive predictive value was 100.0%, and negative predictive value was 75.0% (Figure 3).

### 3.4. Comparison of the Diagnostic Value of Ultrasound and Hysteroscopy in Submucous Myoma of the Uterus

The diagnostic value of ultrasonography and hysteroscopy in submucous myoma of the uterus was compared. Ultrasound and hysteroscopy images in patients with submucous myoma showed uterine cavity protrusion with round or oval, medium and low echo; when the uterine cavity expanded, the tumor protruding into the uterine cavity could be observed. The base width of the myoma, many myomas or giant tumors protruding into the uterine cavity can make the uterine cavity change (Figure 4).

The article "Diagnostic Value of Ultrasonography Combined with Hysteroscopy in Intrauterine Space-Occupying Abnormalities" was published in 2022. Journal: Contrast Media Mol Imaging.

The pathological diagnosis of 27 patients with submucosal myoma of the uterus was confirmed in 33 cases (81.8%). Intrauterine ultrasound was used to diagnose 24 cases of submucous myoma of the uterus, and the diagnostic sensitivity, specificity, accuracy, positive predictive value, and negative predictive value were 88.9%, 50.0%, 81.8%, 88.9%, and 50.0%, respectively. Hysteroscopy was used to diagnose 26 cases of submucous myoma of the uterus, with diagnostic sensitivity of 96.3%, specificity of 83.3%, accuracy of 93.9%, positive predictive value of 96.3%, and negative predictive value of 83.3%. The combined diagnostic sensitivity, specificity, accuracy, positive predictive value, and negative predictive value were 100.0%, 83.3%, 97.0%, 96.4%, and 100.0%, respectively (Figure 5).

### 3.5. Comparison of the Diagnostic Value of Ultrasound and Hysteroscopy in Uterine Fetal Residues

The diagnostic value of ultrasonography and hysteroscopy in uterine fetal residues was compared. The echo in ultrasound and hysteroscopy images of patients with uterine fetal residue was extremely uneven and irregular. Ultrasound can clearly show the location and shape of the residue (Figure 6).

24 cases (72.7%) were confirmed by postoperative pathological diagnosis in 33 patients with uterine fetal residues. 21 cases of uterine fetal residues were diagnosed by intrauterine ultrasound, and the diagnostic sensitivity, specificity, accuracy, positive predictive value, and negative predictive value were 87.5%, 66.7%, 81.8%, 87.5%, and 66.7%, respectively. Hysteroscopy was used to diagnose 22 cases of uterine fetal residues, with diagnostic sensitivity of 91.7%, specificity of 77.8%, accuracy of 87.9%, positive predictive value of 91.7%, and negative predictive value of 77.8%. The sensitivity, specificity, accuracy, positive predictive value, and negative predictive value of combined diagnosis were 95.8%, 88.9%, 93.9%, 95.8%, and 88.9%, respectively (Figure 7).

## 4. Discussion

Intrauterine ultrasound and angiography are the clinical imaging diagnostic methods developed in recent years with extraordinary clinical significance for the diagnosis and treatment of space-occupying abnormalities in the uterine cavity, especially for the pretreatment evaluation of hysteroscopic surgery [19]. Abnormal uterine bleeding and infertility cannot be accurately judged based on history, gynecological examination, and b-ultrasound examination alone [20]. Vaginal ultrasound is characterized by high resolution, good examination effect, easy operation, no trauma, less pain, repeatable, and timely observation of endometrial changes in gynecological diseases, and has high significance for the diagnosis of endometrial problems [21, 22]. Ultrasound is an imaging judgment with some disadvantages and less specificity. Although it can imply submucosal myoma, large endometrial polyps, and intrauterine devices, B-ultrasound has no specificity for indicating small endometrial polyps and submucosal myomas <1.2 cm in diameter. For endometrial lesions with an endometrial thickness <5.1 mm, B-ultrasound observation has a dilemma, or only abnormal echoes in the uterus can be seen. Because there is no method to obtain the final pathological results, the early judgment of endometrial malignant tumors is even more difficult. The traditional method of obtaining pathology is diagnostic curettage. However, diagnostic curettage has certain blindness, limitations, and subjectivity. Small lesions are easily missed, and there is a risk of bleeding. Reports have shown that even experienced gynecologists miss diagnosis rates of traditional curettage by 10.2% to 35.1% [23]. Routine vaginal ultrasonography is a good way to detect the uterus and its adnexa, but it is difficult to detect intrauterine lesions, especially endometrial lesions. SHG is a method developed to noninvasively detect intrauterine lesions. It enhances the specificity of diagnosis of endometrial lesions, can show the location and characteristics of intrauterine lesions, and has high clinical value [24]. The ultrasonic examination method was applied to the diagnosis of various intrauterine space-occupying abnormalities and its diagnostic efficiency was studied. The results showed that the sensitivity, specificity, and accuracy of ultrasonography in the diagnosis of endometrial polyps were 90.0%, 66.7%, and 87.9%, respectively. The sensitivity, specificity, and accuracy of ultrasound in the diagnosis of submucous myoma of the uterus were 88.9%, 50.0%, and 81.8%, respectively. The sensitivity, specificity, and accuracy of ultrasound in the diagnosis of placental residue were 87.5%, 66.7%, and 81.8%, respectively. It was found that the diagnostic efficacy of ultrasound for various types of intrauterine space-occupying abnormalities is still high, which is consistent with the results of previous studies.

The article "Diagnostic Value of Ultrasonography Combined with Hysteroscopy in Intrauterine Space-Occupying Abnormalities" was published in 2022. Journal: Contrast Media Mol Imaging.

In recent years, with the development of hysteroscopy, it can directly observe the shape of the cervix and uterine cavity, and can locate the lesion and sample for biopsy, with unmatched advantages in comparison to B-ultrasound. Hysteroscopy enables observation of the interior of the uterus without damaging the cervix and endometrium. Hysteroscopy is routinely performed when patients with abnormal uterine bleeding do not receive medical treatment or do not achieve the intended treatment. Biopsy-guided treatment is performed based on microscopic findings of suspicious lesions combined with pathological findings [25]. Moreover, hysteroscopic resection can directly treat some diseases, such as intrauterine adhesions, septum resection, submucosal myomectomy, uterine removal, and endometrial polypectomy. In addition, hysteroscopy can directly view the location and type of the device, which combined with B-ultrasound monitoring can significantly improve the success rate of device removal [26]. The study data showed that the effect of ultrasonography combined with hysteroscopy in the diagnosis of endometrial polyps, submucous myoma, and residual uterine conceptuses was higher than that of ultrasonography alone and hysteroscopy alone. Hysteroscopy alone is superior to ultrasonography alone in the diagnosis of endometrial polyps, submucous myomas, and uterine fetal residues. Therefore, hysteroscopy is the most practical way to diagnose the causes in the uterine cavity and cervical canal. The use of hysteroscopy to observe different lesions in the uterine cavity and cervical canal for biopsy makes it easier to determine the location and nature of lesions in the uterine cavity than diagnostic curettage. Compared with other examinations, hysteroscopy has stronger sensitivity and accuracy in the diagnosis of endometrial polyps and submucous myoma, and their differences are statistically significant. Hysteroscopy combined with intrauterine ultrasound can enhance the sensitivity and accuracy of the examination. Vaginal ultrasound is easy to carry out, the patient has no pain, and it is easy to accept. Vaginal ultrasound combined with hysteroscopy has a strong complementary function. The diagnostic effect is accurate and the blindness of the past surgery is reduced. Intrauterine ultrasound and angiography can guide hysteroscopic resection and enhance safety. It can provide clinical data for treatment and provide doctors with treatment methods. Hysteroscopy was applied to the diagnosis of various intrauterine space-occupying abnormalities and its diagnostic efficacy was studied. The results showed that the diagnostic rates of hysteroscopy for endometrial polyps were 96.7%, 66.7%, and 93.9%, respectively. The diagnostic rate of hysteroscopy for submucous myoma of the uterus was 96.3%, 83.3%, and 93.9%, respectively. The diagnosis of placental residue by hysteroscopy was 91.7%, 77.8%, and 87.9%, respectively. It showed hysteroscopy has a good diagnostic effect on various types of intrauterine space-occupying diseases. The efficiency of ultrasound combined with hysteroscopy in the diagnosis of endometrial polyps was 96.7%, 100.0%, 97.0%, 100.0%, and 75.0%, respectively. The diagnostic efficiency of submucous myoma of uterus was 100.0%, 83.3%, 97.0%, 96.4%, and 100.0%, respectively. The diagnostic efficiency of placental residue was 95.8%, 88.9%, 93.9%, 95.8%, and 88.9%, respectively. Therefore, combined diagnosis is more efficient.

The article "Diagnostic Value of Ultrasonography Combined with Hysteroscopy in Intrauterine Space-Occupying Abnormalities" was published in 2022. Journal: Contrast Media Mol Imaging.

## 5. Conclusion

The sensitivity and accuracy of hysteroscopy in the diagnosis of endometrial polyps and submucous myoma are better than that of intrauterine ultrasound, and the combination of them can improve the sensitivity and accuracy of hysteroscopy. Intrauterine ultrasound and angiography can also control hysteroscopic resection, and better enhance the effectiveness. However, the sample size is too small to conduct clinical trials in a single region or small region. More information will be obtained by further increasing the number of cases, which will provide an efficient and direct basis for clinical diagnosis and treatment.

## Figures and Tables

**Figure 1:** (a): Normal uterine cavity by transabdominal ultrasound; (b) normal uterine cavity by transvaginal ultrasound.

**Figure 2:** (a) Comparison of ultrasound; (b) hysteroscopy image in patients with endometrial polyps.

**Figure 3:** Comparison of the diagnostic value of ultrasound and hysteroscopy for endometrial polyps. Se: sensitivity; sp: specificity; ac: accuracy; ppv: positive predictive value; npv: negative predictive value.

**Figure 4:** (a): Ultrasound image of submucous myoma of uterus; (b) hysteroscopy image of submucous myoma of uterus.

**Figure 5:** Comparison of diagnostic value of ultrasound and hysteroscopy for submucous myoma of uterus. se: sensitivity; sp: specificity; ac: accuracy; ppv: positive predictive value; npv: negative predictive value.

**Figure 6:** (a) Ultrasound image of uterine fetal residues; (b) hysteroscopy image of uterine fetal residues.

**Figure 7:** Comparison of the diagnostic value of ultrasound and hysteroscopy for uterine fetal residues. se: sensitivity; sp: specificity; ac: accuracy; ppv: positive predictive value; npv: negative predictive value.

**Table 1:** Comparison of basic data among three groups.

Item	Submucous myoma group	Endometrial polyp group	Placenta residue group	*P*
Sample size	33	33	33	

Age	28.11 ± 1.82	29.26 ± 2.68	25.07 ± 2.54	0.932

History of diabetes				0.819
Yes	9	6	6	
No	24	27	27	

History of smoking				0.707
Yes	10	11	9	
No	23	22	24	

Age of menarche	12.1 ± 1.44	12.8 ± 2.1	11.89 ± 1.33	0.606

First pregnancy				0.511
Yes	12	14	13	
No	21	19	20	

The article "Diagnostic Value of Ultrasonography Combined with Hysteroscopy in Intrauterine Space-Occupying Abnormalities" was published in 2022. Journal: Contrast Media Mol Imaging.

## Data Availability

The data used to support the findings of this study are available from the corresponding author upon request.
